# The Effect of Endoscopy on Patients with Malignant Esophageal Cancer after Medical Treatment and Chemotherapy

**DOI:** 10.1155/2022/7906302

**Published:** 2022-04-09

**Authors:** Yu Liu, Lingqiong Zhao, Xingping Tan, Nana Liu, Teng Long

**Affiliations:** ^1^Department of Oncology, Chongqing General Hospital, University of Chinese Academy of Sciences, Chongqing 400014, China; ^2^Department of Oncology, People's Hospital of Chongqing Hechuan, Chongqing 401520, China; ^3^General Surgery, People's Hospital of Chongqing Hechuan, Chongqing 401520, China

## Abstract

The esophagus is one of the most commonly used parts in a person's life, and its importance is self-evident. With the unhealthy food diet, people are more and more likely to suffer from esophageal cancer, and there is an urgent need for breakthroughs in the treatment of esophageal cancer. This article is aimed at studying the effects of medical treatment and chemotherapy for patients with malignant esophageal cancer. To this end, this article proposes a treatment method based on endoscopy and improves the image imaging of the endoscopy and the image quality of the image and the edge processing of the image. At the same time, this article designs an experiment to conduct statistical analysis of the situation during the treatment process. The experimental results in this article show that the improved treatment method has a 21% increase in success rate compared with the existing treatment method. And the optimized image quality has increased by 27%. It can very well help the attending doctor to improve the efficiency of treatment in the actual treatment process. Its most important contribution is that through the edge optimization and image enhancement processing technology, the success rate of endoscopic treatment has been better improved, and the treatment efficiency has also been improved.

## 1. Introduction

Endoscopic resection can objectively diagnose early esophageal cancer and precancerous lesions and classify them into the disease stage, but the resection technique is a destructive treatment. Because postoperative specimens are not available, early esophageal cancer and precancerous lesions cannot be diagnosed and classified into the disease stage. In order to treat early esophageal cancer and precancerous lesions, it is necessary to develop high-frequency cauterization techniques and research on related factors that affect the clinical prognosis of early esophageal cancer. Now that the more accurate diagnosis of early esophageal cancer and precancerous lesions is established, the prediagnosis system provides the basis for guiding the treatment options of early esophageal cancer and cancer lesions.

The general risk factors for the onset of esophageal cancer are age, smoking, drinking, the intake of pickles, and insufficient trace elements and vitamins. With the improvement of living standards, changes in dietary life, and improvements in sanitation, these are the main reasons that contribute to the suppression of the onset of esophageal cancer, which greatly improves the level of diagnosis and treatment of esophageal cancer. Therefore, the research on effective treatment methods for esophageal cancer is urgent.

With the advent of the era of healthy living, people pay more and more attention to their own bodies, and the improvement of medical standards also guarantees the realization of this demand of the people. Malignant esophageal cancer is one of the most common diseases in the modern era. More and more people are beginning to invest in his treatment research. Tiloke et al. studied the antiproliferative effect of MOE on SNO and determined the cell death mechanism by measuring PS externalization and flow cytometry [1]. In order to solve the uncertainty of whether the clinical staging group (cTNM) of esophageal cancer has the same prognostic significance as the pathological group after simple esophagectomy (pTNM), Rice et al. described the types of cancers and their risks in clinical patients with esophageal cancer from all over the world. The statistical standard is the standard definition of 33 institutions on six continents [2]. Zeng et al. used the latest data collected from the National Central Cancer Registry to provide an estimate of the burden of esophageal cancer in China in 2011. It is based on 177 eligible population-based cancer registries [3]. Feng et al. proposed that Pterocarpus (PTE) is a natural dimethylated resveratrol analogue from blueberries, which is known to have a variety of pharmacological activities, including anticancer properties [4]. Wang et al. proposed to study the definition of planned target volume (PTV) based on four-dimensional computed tomography (4DCT) and traditional PTV definition and the definition of primary thoracic esophageal cancer using asymmetric resection margins. 43 esophageal cancer patients underwent 3DCT and 4DCT simulation scans during free breathing [5]. Otterstatter et al. obtained cancer incidence and mortality from 1986 to 2006 from the Canadian Cancer Registry, the National Cancer Incidence Reporting System, and the Canadian Vital Statistics Death Database [6]. Tan et al. believes that esophageal cancer is composed of esophageal adenocarcinoma and esophageal squamous cell carcinoma. It is one of the most common malignant tumors in the world, especially in southern Iran and China [7]. In Ugo's review of 4,930 resections reported in the Western literature, similar changes are also evident in the literature of Japan and China. The survival rate of the unscreened population has risen from 9% to 23%, and the survival rate of early cancer is as high as 90% [8]. The contents of the mentioned documents are all reasonably designed, and the descriptions of the technology-related content involved in the article are carefully elaborated. However, the experiments carried out are partly based on the experimental results in the theoretical environment, without considering the experimental error brought by the actual operation process and the reliability of the experimental results.

The innovation of this article lies in the theoretical support of the actual operability of ESD technology and the technical support of image enhancement and image edge processing to optimize the medical treatment and chemotherapy of patients with malignant esophageal cancer tumors based on endoscopy. After the improvement, the success rate of the treatment can be effectively improved, and the image quality in the actual operation process has been effectively improved. Compared with the existing system, the improved system has higher recognition sensitivity, the image recognition accuracy rate is also more accurate, and the actual recognition image quality has also been better improved.

## 2. Research Methods

### 2.1. ESD

#### 2.1.1. Definition

ESD is the process of separating the tissue after injection into the submucosal tissue. Choose an appropriate special electrosurgical knife to completely peel off the diseased mucosa and submucosal tissue [9].

#### 2.1.2. ESD Steps

All ESD operations are performed by experienced endoscopy doctors.

Before ESD, narrow-band light observation (NBI) and magnifying endoscopy were used to observe the lesion again to clarify the scope of the lesion. Mark about 5 mm outside the boundary of the target lesion, and after the boundary of the lesion is completely marked, inject the submucosa (glyceride, epinephrine, toluene blue, or a mixture of the solutions). Use the injection needle outside the marked point, and the sign of lifting is positive, during the marking and injection process. According to the various physiological structures of the esophagus and stomach, appropriately adjust the strength of the marking and the depth of injection. After that, incision is made with mucosa around the marking point, and the lesion is slowly peeled off. The incision knife and warm water biopsy forceps are alternately used during the operation. The exposed large blood vessels and the oozing part of the blood are alternately electrically coagulated. Until the lesion is completely peeled off, rinse the wound with water at the same time and observe repeatedly to confirm that there is no bleeding from the wound until the edge of the lesion is completely resected, and the resected lesion is taken out through the mouth [10, 11]. The specific operation steps are shown in Figure 1.

#### 2.1.3. Specimen Processing

Flatten the excised specimen of the endoscope, fix the mucosal surface, and observe and record the relevant data of the specimen (the size and shape of the specimen, the visual field of the lesion). After shooting the film, immerse the specimen in 10 formaldehyde solution [12]. Serial sections were collected every 2 mm and wrapped in paraffin. The steps of endoscopic mucosal dissection are shown in Figure 2.

#### 2.1.4. Pathological Evaluation

Horizontal edge (lateral edge) means that cancer cells remain on the horizontal edge or cannot be distinguished by burning or partial resection that cannot be completely reconstructed. Positive vertical resection edge (undercut edge) means that cancer cells remain on the vertical resection edge or cannot be distinguished due to burning or partial resection that cannot be completely reconstructed. Removal of residual cancer cells on the edge fix the resection specimens of the endoscope; after resection every 2 mm, the sections of the most marginal tissues contain tumor cells. That is to say, the cancer cells are less than 2 mm from the edge of the resection. The so-called total resection refers to the removal of the lesion into one during endoscopy and the collection of one specimen at the same time. Curative resection refers to complete removal of ESD resection specimens without risk of lymph node metastasis. Tumor remains are defined as additional gastrectomy or second endoscopic treatment, and the excised specimens show tumor cells [13].

### 2.2. Research Status of Wireless Endoscopic Image Processing Algorithms

#### 2.2.1. Image Workstation

Various wireless endoscopy devices currently used in clinical practice have corresponding image workstation software. Let us take the software of Israel's Kiven company as an example to introduce. The software is used to support the various stages of wireless endoscopy, including patient login, recorder initialization, data downloading, viewing endoscopic video recordings, and generating inspection reports [14].

#### 2.2.2. Image Enhancement

Image enhancement refers to the preprocessing of wireless endoscopic images to meet the needs of doctors for diagnosis or subsequent processing. It proposes a wireless endoscopic image emphasis method based on diffusion tensor [15]. Experimental results show that the enhanced bleeding image is easily recognized and diagnosed by doctors. In fact, wireless endoscopic images not only affect the uneven brightness distribution but also have disadvantages due to hardware limitations and wireless transmission noise, noise pollution, and blurred edges [16]. Therefore, the wireless endoscope image must be emphasized at the same time as contrast enhancement, image smoothing, and edge sharpening. The image enhancement effect is shown in Figure 3.

#### 2.2.3. Anomaly Detection

Anomaly detection belongs to the highest level of image understanding technology in image processing technology. It is also a field of extensive research and application in wireless endoscope processing technology, but the current research and results in wireless endoscope image disease diagnosis cannot be said to be sufficient [17].

#### 2.2.4. PDE Form of Histogram Equalization

The histogram equalization method is a histogram correction technique with extremely high practical performance. It is suitable for various image imaging conditions, and the direct histogram equalization technology can enhance the contrast of the entire image. However, its enhancement effect is difficult to effectively control, and the image visual effect is relatively rigid and not soft enough. And it is easy to cause the loss of image details [18]. To this end, the following energy functional is established:

(1) $$\begin{array}{c} G\left(I\right)=\frac{1}{2}\int {\left(I\left(p,q\right)-\frac{1}{2}\right)}^{2}dpdq. \end{array}$$

The gradient descent flow of the energy functional of the formula can be expressed as

(2) $$\begin{array}{c} \frac{\partial I\left(p,q,t\right)}{\partial t}=\left[1-\frac{I\left(p,q,t\right)}{I_{\max}}\right]{Α}_{\Omega }-Α\left(I\left(p,q,t\right)\right). \end{array}$$

Equation (2) has a unique steady-state solution:

(3) $$\begin{array}{c} I\left(p,q,\infty \right)=I_{\max}\times E\left(I\right), \end{array}$$

where *E* (*I*) represents the cumulative histogram of the input image. We generalize the histogram equalization operation to the more general arbitrary contrast enhancement operation. Equation (2) can be rewritten as follows:

(4) $$\begin{array}{c} \frac{\partial I\left(p,q,t\right)}{\partial t}=f\left(I\left(p,q,t\right)\right)-I\left(p,q,t\right). \end{array}$$

Traditional image smoothing methods include linear smoothing filters such as mean filtering and Gaussian filtering and statistical sorting filters such as median filtering. The partial differential equation corresponding to the image Gaussian filter is a two-dimensional linear diffusion equation:

(5) $$\begin{array}{c} \frac{\partial I\left(p,q,t\right)}{\partial t}=\mathrm{div}\left(\nabla I\right), \end{array}$$

(6) $$\begin{array}{c} \frac{\partial^{2}I}{\partial x^{2}}+\frac{\partial^{2}I}{\partial y^{2}}=\Delta I, \end{array}$$

where div represents the divergence operator, through the Fourier transformation method, and the solution of the formula can be obtained:

(7) $$\begin{array}{c} I\left(p,q,t\right)=I_{0}\left(p,q\right)*G_{t}\left(p,q\right). \end{array}$$

Add a conductivity term to Equation (5), and it becomes the following form:

(8) $$\begin{array}{c} \frac{\partial I\left(p,q,t\right)}{\partial t}=\mathrm{div}\left[g\left(\left|\nabla I\right|\right)\nabla I\right]. \end{array}$$

Since the initial value problem of the equation may be ill-conditioned, that is, the steady-state solution of the equation does not have continuous dependence on the initial conditions. Therefore, the equation is improved, and the improved regularized diffusion equation is shown in the following equation:

(9) $$\begin{array}{c} \frac{\partial I\left(p,q,t\right)}{\partial t}=\mathrm{div}\left[g\left({\left|\nabla \left(G_{\sigma }*I\right)\right|}^{2}\right)\nabla I\right], \end{array}$$

where *E* (*I*) represents the cumulative histogram of the input image, and div represents the divergence operator.

The use of total variation as the smoothness measure of the image will protect the edges of the image:

(10) $$\begin{array}{c} G\left(I\right)=\frac{1}{2}\lambda \int {\left(I-I_{0}\right)}^{2}dpdq. \end{array}$$

The gradient descent flow that minimizes the energy function is shown in the following equation:

(11) $$\begin{array}{c} \frac{\partial I\left(p,q,t\right)}{\partial t}=\mathrm{div}\left(\frac{\nabla I}{\left|\nabla I\right|}\right)-\lambda \left(I-I_{0}\right). \end{array}$$

In order to alleviate the fragmentation effect of the processing result, the improved total variation denoising model is multiplied by the gradient modulus at the right end of the formula to obtain the following form:

(12) $$\begin{array}{c} \frac{\partial I\left(p,q,t\right)}{\partial t}=\left|\nabla I\right|\mathrm{div}\left(\frac{\nabla I}{\left|\nabla I\right|}\right)-\left|\nabla I\right|\lambda \left(I-I_{0}\right). \end{array}$$

#### 2.2.5. PDE Form with Sharp Edges

Edge sharpening operation and image smoothing are essentially a contradictory process. It corresponds to the reverse diffusion of the image. The most widely used in image sharpening is the Laplacian based on second-order differentiation, which is defined as

(13) $$\begin{array}{c} \nabla^{2}f\left(p,q\right)=\frac{\partial^{2}f}{\partial p^{2}}+\frac{\partial^{2}f}{\partial q^{2}}. \end{array}$$

For discretized two-dimensional images, the following formula can be used as an approximation of the second-order partial differential:

(14) $$\begin{array}{c} \nabla^{2}f=\left[f\left(p+1,q\right)+f\left(p-1,q\right)+f\left(p,q+1\right)+f\left(p,q-1\right)\right]-4f\left(p,q\right). \end{array}$$

To achieve the image sharpening effect, the original image needs to be subtracted from the image processed by the sharpening operator, namely,

(15) $$\begin{array}{c} g\left(p,q\right)=f\left(p,q\right)-\Delta f\left(p,q\right). \end{array}$$

Sharpen the edges of the image by restoring the result of the two-dimensional linear diffusion equation:

(16) $$\begin{array}{c} \frac{\partial I\left(p,q,t\right)}{\partial t}=‐\Delta I. \end{array}$$

The edge detection operator can also adopt more complex forms to enhance the effect of edge detection:

(17) $$\begin{array}{c} \frac{\partial I\left(p,q,t\right)}{\partial t}=-\mathrm{sgn}\left(\Delta I\right)\left|\nabla I\right|. \end{array}$$

From the analysis of the two sections, it is not difficult to see that the smoothing of the image and the sharpening of the edge of the image are essentially a form of diffusion of the image: in the flat area of the image, that is, the area where the gray value does not change much. Perform positive diffusion on the image to smooth the noise points in the image and control the smoothness of the image. In the detailed areas of the image, such as edges, corners, and other shapes, the forward diffusion stops to protect the detailed areas [19, 20]. The specific effect is shown in Figure 4.

#### 2.2.6. Image Enhancement Model

Based on the existing image enhancement methods, we propose an image enhancement scheme based on the image partial differential equation framework. As shown in Equation (18), the framework includes three parts: image contrast enhancement, edge sharpening, and image smoothing [21].

(18) $$\begin{array}{c} \frac{\partial I\left(p,q,t\right)}{\partial t}=\alpha \left(f_{1}\left(I\right)\right)+\beta \left(f_{2}\left(I\right)\right)+\gamma \left(f_{3}\left(I\right)\right). \end{array}$$

Although the improved denoising model avoids the defect of constant image segmentation, the edge protection capability of total variation is also weakened accordingly. We add an edge stop function to weaken the diffusion rate near the edge, so as to achieve the effect of protecting the edge [22]. After the improvement, the fidelity item can be expressed as

(19) $$\begin{array}{c} \frac{\partial I\left(p,q,t\right)}{\partial t}=g\left(\left|\nabla I\right|\right)\left|\nabla I\right|\mathrm{div}\left(\frac{\nabla I}{\left|\nabla I\right|}\right). \end{array}$$

Finally, we proposed the following two-way diffusion equation:

(20) $$\begin{array}{c} f_{2}\left(I\right)=\frac{\partial I\left(p,q,t\right)}{\partial t}=g_{N}I_{NN}+g_{T}I_{TT}. \end{array}$$

In this article, we use the following spread function *g*:

(21) $$\begin{array}{c} g_{N}=\left\{\begin{array}{cc} 0, & \text{if}\;\left|\nabla \left(G_{\sigma }*I\right)\right|>T\\ 1, & \text{otherwise} \end{array}\right., \end{array}$$

(22) $$\begin{array}{c} g_{T}=1-\exp\left(-3.315/{\left(\nabla \left(G_{\sigma }*I\right)/m\right)}^{8}\right). \end{array}$$

Experiments have proved that this value can obtain satisfactory results. Of course, more complex forms can also be used. Adjust the value adaptively according to the size of the gradient near the edge to achieve better results [23].

Compared with images in medicine, the use of machine learning requires a lot of time and data in the early stage, and when there are some more difficult problems, machine learning cannot handle better and may even be missed; so, there is no use and learn to classify.

### 2.3. The Development and Clinical Application of Endoscopy Technology

After more than 100 years of development, digestive endoscopy devices started from rigid endoscopes from the first generation, have been used only for diagnosing digestive tract diseases from the initial stage, and gradually developed to the advanced minimally invasive treatment stage integrating diagnosis and treatment. Compared with surgical operation, endoscopic treatment has less damage to the patient's body, relatively simple technical requirements, faster recovery of patients, less trauma, and a more economical choice. The development process of the endoscope is shown in Figure 5.

Endoscopic resection and endoscopic dissection have been widely carried out in gastroenterology and endoscopic wards of major hospitals. Some secondary hospitals are also actively investing. This endoscopic treatment technique has been widely developed clinically and is mainly used to treat tumors and precancerous lesions that originate in the mucosa and submucosa of the digestive tract. ESD is developed from EMR technology. In addition, after EMR and ESD endoscopic treatment techniques, domestic and foreign scholars have successively proposed more difficult treatment techniques such as endoscopic excavation (ESE), endoscopic tunnel resection, and endoscopic full-thickness resection. It greatly reduces the misdiagnosis rate.

With the continuous maturity of endoscopy technology, innovation and development of endoscopic treatment technology through the natural cavity have been developed. Because it has no incision and no scar after operation, it is now being paid attention to by the majority of endoscopy doctors and patients. In 2009, China established a special NOTES treatment management committee to strictly implement the clinical supervision and application of NOTES. NOTES does not go through a surface approach, which is another milestone in minimally invasive surgery. It is the gospel for obese patients and some patients who cannot tolerate traditional surgery. And because this kind of operation has less interference to the internal environment and less damage to normal tissues and organs, the patient has a relatively fast recovery period and lower cost, and it is more and more accepted by patients. Peroral endoscopic pyloromyotomy is a kind of new NOTES, which is based on ESD technology and transendoscopic tunneling.

Acute upper gastrointestinal bleeding is often caused by acute massive bleeding that causes a sharp decrease in the peripheral blood volume, causing sudden changes in the patient's vital signs. It has become one of the common clinical diseases that threaten the lives of patients. According to global statistics, its annual prevalence and fatality rate are among the best among all acute and critical illnesses. At present, the clinical treatment of acute nonvarice upper gastrointestinal hemorrhage is often performed through endoscopic OTSC metal clip closure. This method of treatment is also considered to be a safe and effective treatment in recent years. However, acute bleeding from esophageal and gastric fundus varices can cause severe bleeding and rapid changes in the condition at the onset of the disease, which often endangers the life of the patient. Therefore, it usually requires painless gastroscopy within 24 hours to clarify the bleeding site and the bleeding situation. According to the performance under the microscope, treatment methods such as endoscopic band ligation, sclerotherapy, and tissue adhesive embolization can be adopted. In addition, a variety of complex endoscopic treatment techniques such as double-gas award enteroscopic polypectomy, hemostasis, stenosis dilation, endoscopic myotomy, acute biliary pancreatitis, combined biliary, and pancreatic drainage can also be used. These endoscopy technologies are clinically emerging in recent years and doctors, and patients are keen on endoscopy. The method of endoscopic metal clip closure is shown in Figure 6.

SMTs of the upper gastrointestinal tract are mainly leiomyomas and GIST, and it is difficult to distinguish GIST from leiomyomas in clinical practice. At present, the most commonly used method is fine needle puncture guided by ultrasound endoscopy. However, the diagnosis rate is not ideal, and the mitotic figures cannot be calculated in pathological specimens obtained by puncture. If SMI's is clinically diagnosed as stromal tumor, its follow-up treatment is controversial. The NCCN guidelines recommend surgical removal of GIST with a diameter of more than 2 cm. If the diameter is less than 2 cm, but EUS finds irregular shape, pockets, ulcers, echogenic foci, or heterogeneity, surgical removal of the lesions is also recommended. The ESMO guidelines recommend that if the histology is confirmed as GIST, surgical resection should be performed.

Endoscopic treatment is a minimally invasive method to remove SMTs in the upper gastrointestinal tract. It is less traumatic, quick to recover, and does not affect the function of the digestive tract. It can not only remove tumors but also provide complete specimens for pathological examination. At present, the main techniques for endoscopic treatment of SMTs derived from the muscularis propria are STER, ESE, and EF. STER is one of the endoscopic tunneling techniques used in clinical practice in the past 4 years. At present, it is mainly used to treat SMTs derived from the esophagus and the lamina propria of mouth. The advantage is that a submucosal tunnel is established at the normal mucosa where the endoscopic space and position are better, the tunnel is separated and extends below the tumor body, and the normal mucosal tissue above the tumor body is preserved. Because the spatial position of the opening is good for the closure of the tablet holder, and after the tunnel is closed, the integrity of the mucosal layer is ensured, and the contact between the wound surface at the tumor bed and the digestive juice and air is isolated. It is more conducive to postoperative recovery and also reduces postoperative complications. However, the tunnel technology itself has its shortcomings. In other words, not all SMTs can be removed using the STER method. Furthermore, endoscopic tunneling technology is one of the most challenging endoscopic technologies at present. It requires a long time of practice, and it takes time to establish the tunnel itself; so, the operation time is longer. Finally, due to the limited space in the tunnel cavity, when the tumor is large, the endoscope cannot be completely removed. Compared with the STE technology, the ESE technology is a direct extension of the ESD technology. It directly cuts the mucosa above the SMTs, then separates the tumor body to complete resection, and finally seals the wound. The advantage is that most upper gastrointestinal SMTs can be treated with this technique. And its operation time is relatively short. The disadvantage is that if the tumor protrudes out of the lumen or the tumor is closely related to the serosal layer, it needs the support of EF technology. In addition, when the tumor is large or the location is special, once perforation occurs, it is difficult to seal the wound with endoscopy, and it is even necessary to suture the wound with thoracoscopy. At the same time, it was found that STER technology has no significant advantages over ESE in terms of complete resection rate and complication rate of upper gastrointestinal submucosal tumors.

Especially in the cardia subgroup, when the tumor is larger (>1.5 cm), the complete resection rate of ESE technique decreases significantly, which may be related to the physiological stenosis of the cardia and the extremely difficult endoscopic operation. Furthermore, the space in the tunnel is limited, and it takes longer to separate the tumor from the tunnel than it takes to separate the tumor after directly incising the mucosa. The main complications of the STER group were subcutaneous emphysema, pneumothorax, and pneumoperitoneum caused by gas entering the interstitial space during the treatment. Due to the use of CO_2_ gas, these complications are within a controllable range. In addition, if the tumor body is found to be closely related to the serosal layer during the separation process, in order to ensure the complete resection of the tumor body, it must be removed together with the serous layer. The integrity of the tunnel is destroyed, and the gas enters the interstitial space from the tunnel inevitably occurs. In the cases where the tumor was completely resected, there was no postoperative gastrointestinal thinness and gastrointestinal infection.

From the experience of endoscopic treatment, the larger the tumor, the longer the operation time of endoscopic resection and the more difficult the operation. The risk of intraoperative perforation, postoperative infection, and delayed bleeding has also increased accordingly. We divided the tumors into subgroups for analysis based on the size of the tumors, and the lesion diameter was 15 mm as the boundary for selection into the group. The results show that the size of the disease has no significant influence on the choice of treatment technique. In other words, the size of the tumor is not a decisive factor in choosing a treatment technique. Especially when the lesions are located in the esophagus-cardia subgroup or the cardia-fundus/high gastric body subgroup, the operation time of the ESE group is shorter than that of the STER group.

Although the intraoperative complications in the STER group were higher, most of them were mild. Statistical analysis shows that we do not need to choose the treatment technique based on the diameter of the lesion but can measure the choice based on multiple factors such as the location of the lesion, the operation time, the complications, and the difficulty of the operation. For this reason, we recommend the STER method for SMTs with larger diameters (diameter > 1.5 cm) at the EGJ site, especially for lesions with irregular shapes, because of its high complete resection rate and low complication rate (except for the complications of gas entering the interstitial space). For smaller SMT (1.5 cm diameter), we recommend ESE treatment, because of its relatively short operation time, high complete resection rate, and relatively few complications.

## 3. Questionnaire Experiment

### 3.1. Lesion Characteristics

This experiment randomized investigation 126 conducted experimental investigations for patients. Before the experiment, first conduct a statistical investigation on the experimental objects. The specific information is shown in Table 1.

From the table, we can see that there are 60 cases in the ESD group, including 42 males and 18 females; the age is 57-71 years old. There were 4 cases in the upper segment, 46 cases in the middle segment, and 10 cases in the lower segment; there were 66 cases in the surgical group. Among them, there were 42 males and 18 females, aged 67-55 years, 10 cases in the upper segment, 44 cases in the middle segment, and 12 cases in the lower segment. It can be seen that in the ESD group, most of the cases are distributed in the middle section, and this is also the case in surgical operations. Therefore, we should focus on the middle section in the later experimental research. And the two groups of patients were not statistically significant in terms of age and gender (*p* > 0.05). At the same time, this experiment carried out experimental statistics on the resection rate at different degrees, and the specific conditions are shown in Table 2.

From the table, we can see that in the ESD treatment group, the en bloc resection rate is 100%. In the surgical treatment group, the en bloc resection rate was also 100%. In the ESD treatment group, the probability of complete resection rate was 96.6%. The complete resection rate in the surgical treatment group was 96.9%, which was higher than the 96.6% in the ESD treatment group. In the ESD treatment group, the curative resection rate was 96.6%. In the surgical treatment group, the curative resection rate was 96.9%. At the same time, this experiment counts the relevant time of the experiment and counts the integration of its operation time and hospitalization time. The specific data is shown in Table 3.

From the table, we can see that the operation time of the ESD treatment group was 128.14 ± 35.61 minutes, and the hospital stay was 15.64 ± 6.23 days. In the surgical treatment group, the operation time was 321.49 ± 98.35, and the hospital stay was 31.26 ± 11.36 days. In terms of time comparison, it can be seen that the time of the surgical treatment group is much longer than that of the ESD treatment group, no matter in the operation time or the number of days of hospitalization. At the same time, the operation time and hospitalization days of the two groups were statistically significant (*p* < 0.05). The operation time and hospital stay of the surgical group were longer. At the same time, in order to explore the problems of complications and recurrence after and during the operation, this article counts the complications during the operation. The statistics are shown in Table 4.

From the table, we can see that in the ESD treatment group, the probability of recurrence is 3.33%, the probability of bleeding is 3.33%, the probability of perforation is 3.33%, the probability of stenosis is 6.67%, and there is no infection. In the surgical treatment group, there was no recurrence, the probability of bleeding was 24.24%, there was a probability of no perforation, the probability of stenosis was 9.09%, and the probability of infection was 9.09%. At the same time, we design here to conduct statistics on the postoperative quality of life of patients through review of endoscopy, telephone follow-up, and outpatient review. The statistics are shown in Table 5.

From the data in the table, we can see that in the results of the review endoscopy and telephone follow-up, patients with gastrointestinal symptoms mainly have the following symptoms: abdominal distension, acid reflux, and heartburn. The endoscopic manifestations mainly have the following three symptoms: whether the anastomosis is healed, whether there is erosion, and whether there is stenosis. Statistical analysis showed that the chi-square value was *p* < 0.001, and the difference was statistically significant. The ESD treatment group was better than the surgical operation group.

## 4. Result Analysis

### 4.1. Analysis of Follow-Up Results and Clinical Characteristics of Patients with Noncurable Resection of Early Malignant Esophageal Cancer Tumors and Patients Treated with Endoscopy

In order to ensure the accuracy and reliability of the follow-up results, the patients surveyed in this experiment were conducted in accordance with standards. It is based on a certain degree of follow-up, investigating the quality of life, evaluating using a scoring scale for scoring, and at the same time conducting follow-up in combination with telephone to ensure the diversity of follow-up. At the same time, a questionnaire survey experiment was carried out for all early patients, and statistics were collected on the conditions and emotional problems of the patients during the investigation and follow-up. According to the statistical results, the results are shown in Figure 7:

At the same time, the clinical characteristics of early esophageal cancer patients with cured/noncured resection were compared and analyzed. The comparison result is shown in Figure 8.

From the two figures, we can see that the treatment of nausea in patients with early noncurative resection is slightly due to the low level of patients treated under endoscopy. The scores of the rest of the adverse conditions are higher than the treatment scores based on patients under endoscopy. The highest nausea score of early patients was 1.6, and the lowest was 0.8, which was lower than the highest 2.0 and lowest 0.6 based on endoscopic treatment. Among the adverse symptoms of decreased appetite, the early score is the highest 3.1 and the lowest 0.5, which is higher than the highest 1.4 and the lowest 0.8 based on endoscopic treatment. Among the adverse symptoms of weight loss, the early score is the highest 2.3 and the lowest 0.5, which is higher than the highest 1.6 and the lowest 0.8 based on endoscopic treatment. Among the adverse symptoms of nervousness, the early score is 3.9 at the highest and 0.9 at the lowest, which is higher than the highest 1.8 and the lowest 0.8 based on endoscopic treatment. In terms of clinical features, the early cure of esophageal cancer has less impact on gender. The overall age is higher than the clinical characteristics of patients with noncurable resection. In terms of tumor diameter, there is little difference between the two, but noncurative resection is more likely to be affected by the tumor site. In summary, it can be seen that nausea can occur in treatment based on endoscopic treatment, which is slightly higher than that of early treatment. Other symptoms are obviously better than early treatment.

### 4.2. Comparison of 3-Year Survival Rate between Two Groups of Patients with Different Lymph Node Metastases

A stratified analysis of the independent factors affecting the prognosis of the entire group of patients showed that the 3-year survival rate of pN0 patients in the long-diameter group and the short-diameter group was not statistically significant (*p* > 0.05). The 3-year survival rate of pN1 patients in the long-diameter group and the short-diameter group was not statistically significant (*p* > 0.05). The specific situation is shown in Figure 9.

### 4.3. Factors Affecting the Prognosis of the Whole Group of Patients

According to univariate analysis, the position of the upper edge of the tumor under the endoscope, the length of the tumor under the endoscope, the vascular tumor thrombus, the number of lymph node metastases, and the pathological type were found. Further analysis based on the COX proportional hazard model showed that endoscopic tumor length, vascular tumor thrombus, and number of lymph node metastases were independent factors affecting the prognosis of the entire group of patients. The risk model analysis is shown in Figure 10.

It can be seen that the length of the tumor is a factor that cannot be ignored. It is closely related to other factors such as the depth of esophageal cancer tumor invasion and lymph node metastasis. As the length of the tumor increases, the number of lymph node metastases increases. The longer the tumor length, the deeper the invasion and the more extensive the lymph node metastasis.

## 5. Conclusion

The main research content of this article is based on the effects of medical treatment and chemotherapy in patients with malignant esophageal cancer tumors under endoscopy. For endoscopic treatment, this article first analyzes it in the method section. This article has a detailed understanding of its treatment methods and treatment process. There is also this article to optimize the imaging of the endoscope. This paper proposes edge optimization and methods for image enhancement processing. The experimental part also used questionnaires to understand the patient's response during the operation and after the operation. By comparing the advantages of endoscopic treatment, it is finally analyzed. The analysis results show that the success rate of endoscopic treatment has increased by 21% compared with previous methods, and the optimized image quality has increased by 27%. It greatly improves the difficulty of treatment and also improves the efficiency of treatment. A suggestion here is to add denoising and noise reduction processing in image processing, which can make the processed image clearer.

## Figures and Tables

**Figure 1:** ESD operation steps.

**Figure 2:** The process of endoscopic mucosal dissection.

**Figure 3:** Image enhancement effect.

**Figure 4:** Comparison of edge processing effects.

**Figure 5:** The development history of endoscopy.

**Figure 6:** Endoscopic metal clip closure operation.

**Figure 7:** Comparison of follow-up results of patients with noncurable resection and endoscopic treatment.

**Figure 8:** Comparison of clinical characteristics of early esophageal cancer patients with cured/noncurable resection.

**Figure 9:** Comparison of survival rates of different lymph node metastases.

**Figure 10:** Analysis of prognostic factors affecting the whole group of patients.

**Table 1:** Survey statistics of experimental subjects.

Basic parameters	ESD treatment group	Surgical treatment	*p* value
Number of cases	60	66	0.468
Age	64 ± 7	61 ± 6	0.272
Gender: male female	42/18	42/24	0.769
Upper section	4	10	0.366
Middle section	46	44	0.523
Next paragraph	10	12	0.379

**Table 2:** Composition ratio of different resection degrees.

Basic parameters	ESD treatment group	Surgical treatment	*p* value
En bloc resection rate	(60/60) 100%	(66/66) 100%	—
Complete resection rate	(58/60) 96.6%	(64/66) 96.9%	0.923
Curative resection rate	(58/60) 96.6%	(64/66) 96.9%	0.647

**Table 3:** Relevant time of the patient's surgery.

Basic parameters	ESD treatment group	Surgical treatment	*p* value
Operation time (minutes)	128.14 ± 35.61	321.49 ± 98.35	<0.001
Hospitalization time (days)	15.64 ± 6.23	31.26 ± 11.36	<0.001

**Table 4:** Statistics of postoperative complications and recurrence of patients.

Basic parameters	ESD treatment group	Surgical treatment	*p* value
Relapse	(2/60) 3.33%	Without	—
Bleeding	(2/60) 3.33%	(16/66) 24.24%	<0.01
Perforation	(2/60) 3.33%	Without	—
Narrow	(4/60) 6.67%	(6/66) 9.09%	0.127
Infect	Without	(6/66) 9.09%	—

**Table 5:** Postoperative quality of life of patients.

Basic symptoms	ESD treatment group	Surgical treatment	*p* value
Digestive symptoms			
Nausea	6	24	<0.05
Vomit	2	20	<0.05
Acid reflux	10	40	<0.05
Heartburn	12	44	<0.05
Bloating	6	10	>0.05
Decreased appetite	4	16	<0.05
Weight loss	4	8	>0.05
Endoscopic performance			
Anastomotic hyperemia	2	20	<0.05
Anastomotic erosion	4	10	>0.05
Narrow	2	0	>0.05

## Data Availability

The data that support the findings of this study are available from the corresponding authors upon reasonable request.
